This article has been retracted.

# Histological Classification and Invasion Prediction of Thymoma by Machine Learning-Based Computed Tomography Imaging

**DOI:** 10.1155/2022/4594757

**Published:** 2022-08-05

**Authors:** Danfeng Wang, Yiwei Zhang, Bingli Li, Qiaowei Zhuang, Xiaoqin Zhang, Daiying Lin

**Affiliations:** Department of Radiology, Shantou Central Hospital, Shantou 515031, Guangdong, China

## Abstract

**Purpose:**

The values of machine learning-based computed tomography (CT) imaging in histological classification and invasion prediction of thymoma were investigated.

**Methods:**

181 patients diagnosed with thymoma by surgery or biopsy in Shantou Central Hospital between February 2017 and March 2022 were selected. According to the concept of simplified histological classification and the latest histological classification by the WHO, thymoma was divided into two groups, including low-risk (types A, AB, B1, and metaplastic type) and high-risk groups (types B2 and B3). CT images were reconstructed by filtering back projection (FBP) algorithm. CT image features were collected for statistical analysis.

**Results:**

The main symptoms of patients diagnosed with thymoma included respiratory tract infection, chest distress and shortness of breath, and chest pain. 35.91% of them suffered from complicated myasthenia gravis. Tumor size and position in low-risk and high-risk groups showed no statistical significance (*P* > 0.05). Tumor morphology and boundary between the two groups suggested statistical difference (*P* < 0.05). Whether tumor invaded adjacent tissues was apparently correlated with simplified histological classification (*P* < 0.01). The sensitivity and specificity of CT images for the invasion of mediastinal pleura or pericardium were around 90% and negative predictive values both reached above 95%. Those of the CT images for lung invasion were over 80%. The negative and positive predictive values were 93.54% and 63.82%, respectively. Those of the CT images for blood vessel invasion were 67.32% and 97.93%. The negative and positive predictive values were 98.21% and 83%, respectively.

**Conclusion:**

The machine learning-based CT image had significant values in the prediction of different histological classification and even invasion level.

## 1. Introduction

Thymoma is a malignant tumor caused by the lesions at human thymus site [1, 2]. Thymus gland is located behind the sternum and next to the heart and is one of the lymphatic organs in human body [3]. Its main function is to produce leukocyte to resist the invasion of foreign pathogens. According to the current studies on thymoma, most of them is malignant. However, it does not grow quickly with low malignancy. Hence, patients can still live for a long time even if suffering from this disease [4]. At present, the pathogenesis of thymoma is still unclear. Medical community generally believes that some risk factors [5], such as radiation, chemical substance, and genetic factors, increase the risk of suffering from this disease. In the early stage of thymoma, most patients obviously suffer from chest discomfort and pain, and a few patients suffer from weight loss, night sweating, respiratory discomfort, or dyspnea. As tumors grow, superior vena cava obstruction occurs. After 2015, the WHO updated the view of histological classification of thymic epithelial neoplasms [6]. All types of thymomas were considered as malignant tumors (except for micronodular thymoma with lymphoid stroma (MNT) and microscopic thymoma). Thymoma is divided into the following subtypes, including type A, type AB, type B1, type B2, type B3, a few nontypical type A, metaplastic type, and sclerotic type.

Surgical treatment is the preferred choice of the clinical treatment for patients with thymoma [7, 8]. The preoperative diagnostic result has a significant impact on the treatment plan for patients. Imaging examination plays an important role in preoperative diagnosis. So far, computed tomography (CT) examination is still the most widely used method during the diagnosis of thymoma. In clinical practice, CT examination can be adopted to predict the histological classification of thymoma [9, 10].

Because of the rapid innovation and development of multi-slice spiral CT scanning technology, CT plain scan is the most frequently used examination method for early chest screening [11]. Nonetheless, the CT examination itself has some disadvantages [12]. For instance, the radiation dose it uses is much more than routine X-ray examination compared with traditional X-ray examination. Hence, the clinical use of CT diagnosis shows certain limitations. The reduction in radiation dose will make images become noisy and image quality much lower [13], which is far from meeting the needs of clinical diagnosis. A new generation of filtering back projection (FBP) algorithm can greatly reduce image noise and improve image quality with only a small amount of dose [14]. In the research, the histological classification and invasion prediction of thymoma by iterative algorithm-based CT images were investigated.

## 2. Methods

### 2.1. Research Objects and Grouping

A total of 181 patients diagnosed with thymoma by surgery or biopsy in Shantou Central Hospital between February 2017 and March 2022 were selected as the research objects. The complete clinical, pathological, and CT imaging data on patients were summarized. Among 181 included patients, there were 73 male patients and 108 female patients aged between 10 and 81. According to the concept of simplified histological classification put forward by Jeong et al. [15] and the latest histological classification by the WHO, all patients were divided into two groups, including the low-risk group (type A, type B, type B1, and metaplastic type) and the high-risk group (type B2 and type B3). Two experienced diagnostic physicians were selected to observe, identify, and analyze patients' images. The detailed information about patients were not told to them in advance, while they were informed of thymoma as the results in advance without specific histological classification. If there was a disagreement over the final analysis results between the two physicians, a unified conclusion was reached through discussion. The CT images were analyzed from the following aspects, such as tumor size, position, morphology, boundary [16–18], uniformity of density, and the presence of calcification, cystic necrosis, peripheral invasion, and distant metastasis. Besides, patient's clinical manifestations and laboratory examination results were collected for statistical analysis. The correlation between machine learning-based CT image features and histological classification was evaluated. The implementation of this research had been approved by Shantou Central Hospital Medical Ethics Committee. In addition, patients and their family members had understood research contents and methods and agreed to sign corresponding informed consent forms.

The inclusion criteria were as follows:

- Patients diagnosed with thymoma by pathological diagnosis
- Patients whose nodal diameter ranged between 10 mm and 30 mm
- Patients with high-quality CT images and observable imaging signs
- Patients without receiving chemotherapy or radiotherapy [19, 20]
- Patients who agreed to and were willing to cooperate with imaging diagnosis

The exclusion criteria were as follows:

- Patients with other complicated system diseases or serious infectious disease
- Patients with incomplete clinical data and information
- Patients allergic to contrast agents

### 2.2. The CT Scan of Patients' Chest

Chest CT scan and whole-body low-dose CT examination were conducted on 181 patients (Siemens Somatom Emotion 16-slice spiral CT scanner was used). The scan ranged from the apex of the lung to the costophrenic angle. The scan for a few patients with cervical ectopic thymoma ranged from the inferior margin of hyoid bone to the superior margin of aortic arch [21]. The scan parameters were set as follows: tube voltage was 120 kV, auto-milliampere matrix was 512 × 512, the rotation time was 0.6 s, scan slice thickness was 5 mm, and image slice thickness was 1.25 mm. The mediastinum window parameters were set as follows: window width was 350HU and window level was 50HU. The nonionic contrast medium used for enhanced scan was Omnipague (the concentration was 300 mg/mL) and the dose was 1.5 mL/kg (60 to 80 mL for neck). During the enhanced scan, a high-pressure syringe was used for intravenous bolus injection at a flow rate of 2.5 mL/s.

### 2.3. Histological Classification

In 1999, thymoma was divided into the following 6 types by the WHO, including A, AB, B1, B2, B3, and type C (type C represented thymic carcinoma). Because thymic carcinoma was featured with differentiation model, absence of organoid structures, and significant cellular atypia, another classification was carried out by the WHO in 2004. Thymic carcinoma was not classified with other types of thymomas. In 2014, thymoma classification was redefined by the WHO. Thymoma was defined as a type of malignant tumor. Besides, thymoma with lymphoid stromal micronodules was not regarded as benign tumor any more. The concept of mixed thymoma was not used any longer and replaced with the concept of mixed thymic carcinoma. Meanwhile, the differences among various subtypes were explained in detail. The methods for identifying various histological classifications of thymoma were described as follows: Type A consisted of most fusiform or oval epithelial cells lacking nuclear heterotropy and a few T lymphocyte lacking terminal deoxynucleotidyl transferase (TDT) positive. Type AB consisted mainly of fusiform or oval epithelial cells lacking nuclear heterotropy and T lymphocyte with TDT positive in focal or total range. Type B1 thymoma consisted of a great number of immature T lymphocyte, medullary differentiation area, and a small proportion of nontufted epithelial cells. Type B2 thymoma consisted of considerable immature T lymphocyte and many pleomorphic atypical epithelial cells. Type B3 thymoma consisted of a small proportion of mature T lymphocyte and numerous pleomorphic mild to moderate atypia epithelial cells. Metaplastic type thymoma was a biphasic low-level malignant tumor consisting of intertwining epithelial cells and fasciculate fusiform cells [22]. In 2004, Jeong divided 5 types and thymic carcinoma into the low-risk group (type A, type AB, and type B1), the high-risk group (type B2 and type B3), and the thymic carcinoma group. This method was widely supported and applied. Because the morphological difference between metaplastic type thymoma and type A was not very significant, patient thymoma was divided into two groups based on the reference to the simplified histological classification by Jeong et al. including the low-risk group (type A, atypical type A, type AB, type B1, and metaplastic type) and the high-risk group (type B2 and type B3).

### 2.4. Filtering Back Projection (FBP) Algorithm

The first step of FBP is that the projected data are filtered. Next, the reconstructed images are obtained from the projected data by back projection operation [23–25]. For the specific slices in one of the layers of the reconstructed object, the attenuation coefficients of the ray corresponding to all points on the loading surface can be reconstructed by projection values [26, 27]. *R*_0_ refers to the velocity before the ray passes through an object, *R* denotes the intensity after the ray passes through an object, and *φ* (*x*, *y*) represents the linear attenuation index of substance to ray at (*x*, *y*). Monochromatic ray is taken as the example, and equation (1) is shown as follows:

(1) $$\begin{array}{c} R=R_{0}\exp\left(-\int \varphi \left(x,y\right)\text{d}L.\right. \end{array}$$

The logarithm is taken on both sides to generate

(2) $$\begin{array}{c} \int \varphi \left(x,y\right)\text{d}L=\ln\;R_{0}-\ln\;R. \end{array}$$

Equation (3) is expressed as follows:

(3) $$\begin{array}{c} Q\left(t,\theta \right)=\int \varphi \left(x,y\right)\text{d}L. \end{array}$$

In equation (3), *q* (*t*, *θ*) is called as the line integral of the function *φ* (*x*, *y*) along the ray *L* (*t*, *θ*) or projection data. The ray *L* (*t*, *θ*) is called the projection line, which meets the relationship of *x*cos*θ* + ysin*θ* = *t*.

The two-dimensional Fourier transform of the image to be reconstructed *φ* (*x*, *y*) is set to be *F*(*v*_1_, *v*_2_) and the Fourier transform of projection data *q* (*t*, *θ*) is set to be *q* (*ρ*, *θ*). The following equation is obtained based on projection theorem:

(4) $$\begin{array}{c} \varphi \left(x,y\right)=\int_{0}^{ƛ}\text{d}\theta \int_{-\infty }^{\infty }Q\left(\rho ,\theta \right)e^{i2\rho }\left|\rho \right|\text{d}\rho . \end{array}$$

Equation (4) can be transformed into the discrete form

(5) $$\begin{array}{c} \varphi \left(x,y\right)=\frac{d\cdot \Delta \theta }{2ƛ}\sum_{s=0}^{n-1}\sum_{h=-\infty }^{\infty }q\left(t_{h},\theta_{s}\right)\times G\left(x\;\cos\;\theta_{s}+y\;\sin\;\theta_{s}-t_{h}\right). \end{array}$$

In equation (5), *θ*_*s*_=*s* · △*θ*, *n* refers to the total number of projection, *G* denotes filtering function, *th* = *hd*, *h* = 0,+1, +2,… represents the number of rays, and *d* refers to ray spacing. In terms of parallel beam, the two-dimensional distribution of attenuation index of the original object *φ* (*x*, *y*) can be acquired by the projection data in the whole space *q* (*t*, *θ*). FBP algorithm is based mainly on noise reduction in front and rear projection domains. Its principle frame is displayed in Figure 1.

### 2.5. Evaluation Indexes

Specificity and sensitivity were adopted to assess the diagnostic effects of three different diagnosis methods on thymoma in the research. The calculation methods were expressed as follows:

(6) $$\begin{array}{c} \text{specificity}=\frac{b}{c+b}, \end{array}$$

(7) $$\begin{array}{c} \text{sensitivity}=\frac{a}{d+a}. \end{array}$$

In equations (6) and (7), *a* referred to true positive (the diagnostic result was positive, and the actual result was positive), *b* indicated true negative (the diagnostic result was negative, and the actual result was negative), *c* suggested false positive (the diagnostic result was positive, and the actual result was negative), and *d* represented false negative (the actual result was positive, and the diagnostic result was negative).

### 2.6. Statistical Methods

All research data were analyzed with SPSS 24.0 statistical software. The simplification of the long and short diameters of tumor cross section, enhanced plain CT value, and age between groups was performed by one-factor analysis of variance. Tumor morphology, position, calcification, calcification type, uniformity of density, enhancement level, peripheral invasion, and distant metastasis were analyzed with the chi-square test. *P* < 0.05 indicated statistical significance. *P* ≥ 0.05 showed no statistical significance.

## 3. Results

### 3.1. Patient Basic Information

The statistical results of basic information about the patients in the two groups were displayed in Table 1 and Figure 2. It was found that there were 136 patients in the low-risk group and 45 patients in the high-risk group. The proportions of male patients in the two groups were 22.10% and 18.23%, while those of female patients in the two groups were 27.63% and 32.04%. The difference in gender ratio between the patients in the two groups demonstrated no statistical significance (*P* > 0.05). Besides, the proportions of patients at different age groups in the two groups all showed no statistical significance (*P* > 0.05). The proportions of the patients with cystic necrosis in the low-risk group and the high-risk group amounted to 6.08% and 7.18%, respectively.

### 3.2. Histological Classification

According to the histological classification by the WHO, type A patients accounted for 4.41%, including males accounting for 1.10% and females accounting for 3.31% among 181 patients. Type AB patients accounted for 13.26%, including males accounting for 5.52% and females accounting for 7.72%. The proportion of type B1 patients reached 8.29%, including males for 2.21% and females for 6.08%. Besides, the proportion of metaplastic type patients amounted to 49.17%, including males for 20.99% and females for 28.18%. B2 patients accounted for 16.02%, including males for 6.08% and females for 9.94%. B3 type patients accounted for 8.82%, including males and females both for 4.41%, as shown in Figure 3 and Table 2. According to the simplified histological grouping method, the proportion of the patients (Type A, type AB, type B1, and metaplastic type) in the low-risk group was 75.16%, including males for 29.84% and females for 45.32%. The patients (Types B2 and B3) in the high-risk group accounted for 24.84%, including males for 10.49% and females for 14.35%.

### 3.3. Correlation between Clinical Symptoms and Histological Classification

Among 181 patients, both clinical symptoms and simplified histological classification revealed no statistical significance (*P* > 0.05). 67 patients (37.02%) were diagnosed with tumor by physical examination or by chance. 18 patients (9.94%) with thymoma suffered from respiratory tract infection. 14 patients (7.73%) suffered from chest distress and shortness of breath. 9 patients (4.97%) suffered from chest pain. 2 patients (1.10%) suffered from palpitation. 3 patients (1.66%) suffered from hoarse voice. 3 patients (1.66%) visited the hospital for fever. A total of 65 patients (35.91%) suffered from paraneoplastic syndrome of myasthenia gravis (MG), as shown in Table 3. In addition, 3 patients (1.66%) suffered from pure red cell aplasia (PRCA) and 2 (1.10%) suffered from rheumatic arthritis.

### 3.4. CT Signs of All Subtypes of Thymoma

As displayed in Figure 4, Figure 4(a) showed patient thymoma in the low-risk group. Tumor shape looked similar to a round and regular. Besides, tumor edge was smooth. Figure 4(b) displays the thymoma CT image of a female patient aged 35. The lump was located at the right anterior superior mediastinum. Tumor shape was irregular, the edge was not very smooth, and the adjacent adipose layer disappeared.

### 3.5. Correlation between the CT Image Features and Histological Classification

#### 3.5.1. Tumor Size and Position

The long diameters of the maximum tumor cross sections of simplified classification in the low-risk group and the high-risk group were 5.28 ± 2.11 cm and 5.02 ± 2.02 cm (*P*=0.258), respectively. The short diameters of the corresponding slices in the low-risk group and the high-risk group were 3.70 ± 1.53 cm and 3.49 ± 1.52 cm (*P*=0.300), respectively. Hence, there was no statistical significance in tumor short and long diameters between the low-risk group and the high-risk group.

#### 3.5.2. Tumor Shape and Boundary

Tumors in the low-risk group tended to be round or elliptical, while tumor shape in the high-risk group tended to be irregular. The tumor shapes of the two groups showed statistical difference (*P* < 0.05).

#### 3.5.3. Tumor Invasion and Metastasis

Thymoma might invade peripheral lung tissues, pericardium, pleura, and aorta. The invasion of adjacent tissues by thymoma occurred among a total of 12 patients, including 4 cases in the low-risk group and 8 in the high-risk group. Among 162 patients, no invasion of adjacent tissues by thymoma was found, including 125 cases in the low-risk group and 37 in the high-risk group. Whether tumors invaded adjacent tissues was significantly correlated with simplified histological classification (*P*=0.008 < 0.01), which suggested that thymoma in the high-risk group was more likely to invade adjacent tissues.

The correlation between the CT image features and histological classification is illustrated in Figure 5.

### 3.6. Predictive Analysis of Thymoma Invasion by CT Performance

As illustrated in Figure 6, the sensitivity and specificity of CT for thymoma invasion of mediastinal pleura or pericardium were around 90% and negative predictive values both reached over 95%. The sensitivity and specificity of the CT scan for lung invasion were higher than 80%. The negative and positive predictive values amounted to 93.54% and 63.82%, respectively. In addition, the sensitivity, specificity, negative predictive value, and positive predictive value for blood vessel invasion were 67.32%, 97.93%, 98.21%, and 83%, respectively.

## 4. Discussion

Thymoma is a type of low-level malignant tumor appearing in thymic epithelium. However, it is usually volatile and invades adjacent tissues. Hence, surgical treatment is a commonly used clinical method for thymoma. Therefore, preoperative accurate assessment of disease by CT examination has a significant impact on the selection of clinical surgical plans and therapeutic effect [28].

During the clinical diagnosis and treatment, about 40% of patients with thymoma does not suffer from obvious symptoms, most of which are detected by physical examination. When the disease progresses to a certain stage, patients diagnosed with thymoma usually suffer from one or more of the following symptoms, including cough, disturbance in respiration, chest discomfort, palpitation, and hoarse voice [29]. All included patients suffered mainly from the following symptoms, including cough, disturbance in respiration, and chest discomfort. In most cases, the patients with thymoma suffer from MG. According to relevant literature, about 30% of patients with thymoma suffered from MG, especially among young people [30]. In this research, 35.91% of patients were diagnosed with MG, which was higher than that in relevant studies. The reason might be the young age of the selected samples. The final results of the study on the correlation between the CT image features and histological classification indicated that there was no statistical significance in tumor size and position between the low-risk group and the high-risk group (*P* > 0.05). Tumor shape and boundary showed statistical differences between the low-risk group and the high-risk group (*P* < 0.05). Besides, whether tumors invaded adjacent tissues was apparently correlated with histological classification (*P* < 0.01). The experimental results in this research demonstrated that the invasion of adjacent tissues in the high-risk group was more frequent than that in the low-risk group. Therefore, thymoma in the high-risk group was featured with the invasion of adjacent tissues. The results of the predictive analysis of thymoma invasion by CT performance suggested that the sensitivity and specificity of machine learning-based CT for thymoma invasion of mediastinal pleura or pericardium were both around 90%. Besides, negative predictive values were both over 95%. Hence, the results of machine learning-based CT examination could provide useful reference and basis for thymoma patients who needed clinical surgical treatment and help physicians better determine whether tumors could be resected, tumor complete resection rate, and whether adjuvant treatment was required. As a result, surgical success rate could be improved to help patients get rid of disease more quickly. Both the sensitivity and specificity of machine learning-based CT for lung invasion were higher than 80% and negative predictive value amounted to 93.54%. Hence, it could be viewed as a valuable preoperative reference for physicians to evaluate lung invasion among patients. Its positive predictive value was 63.82%, which might be associated with the small sample size selected in the research. The reason needed to be further investigated. The sensitivity of CT examination for blood vessel invasion was 67.32%, which was also related to the small number of the patients with blood vessel invasion. The specificity of CT examination for blood vessel invasion and its negative predictive value reached 97.93% and 98.21%, respectively. Hence, machine learning-based CT examination showed great values in identifying blood vessel invasion. According to the research results, machine learning-based CT examination could make a good judgment on the invasiveness of thymoma. The application of machine learning-based CT examination provided more appropriate surgical plans for patients who needed surgical treatment and improved tumor resection rate as well as integrity and prognostic effects on patients to help patients recover more quickly.

## 5. Conclusion

The imaging manifestations of thymomas in the low-risk group were mostly round-like or elliptical with clear boundaries and obvious enhancement after enhancement. Cystic necrosis was likely to occur among thymomas in the high-risk group and most of them invaded adjacent tissues. Type A thymoma was tended to be limited and uniform small lumps, while central dotted and clustered calcification and peripheral invasion were more likely to appear in Type B3 thymoma. Machine learning-based CT imaging showed a significant value in the prediction of different histological classifications and even the invasion levels of thymoma.

## Figures and Tables

**Figure 1:** The FBP algorithm.

**Figure 2:** Patient basic information. (a) The treatment methods for patients and (b) whether focal calcification occurred.

**Figure 3:** Histological classification of 181 cases with thymoma.

**Figure 4:** CT images of patients with thymoma. (a, b) The CT images of two different patients.

**Figure 5:** Correlation between the CT image features and histological classification. (a) Tumor shape, (b) tumor position, (c) whether tumor edge was clear, and (d) whether there was peripheral invasion.

**Figure 6:** Predictive analysis of thymoma invasion by CT performance. (a) Positive predictive value, (b) negative predicative value, (c) sensitivity, and (d) specificity.

**Table 1:** Basic information about the patients in the two groups.

Items	Types	Patient proportion (%)	
		Low-risk group	High-risk group
Gender	Male	53 (29.28%)	20 (11.05%)
	Female	83 (45.86%)	25 (13.81%)

Age	Average age	48 ± 9.81	51 ± 11.39

Lesion cystic necrosis	Yes	11 (6.08%)	13 (7.18%)
	No	79 (43.65%)	78 (43.09%)

**Table 2:** Gender ratio of 181 cases with thymoma.

Gender	Type A	Type AB	Type B1	Metaplastic type	Type B2	Type B3
Male	2 (1.10%)	10 (5.53%)	4 (2.21%)	38 (20.99%)	11 (6.08%)	8 (4.41%)
Female	6 (3.32%)	14 (7.73%)	11 (6.08%)	51 (28.18%)	18 (9.94%)	8 (4.41%)
Total	8 (4.42%)	24 (13.26%)	15 (8.29%)	89 (49.17%)	29 (16.02%)	16 (8.82%)

**Table 3:** Correlation between clinical symptoms and histological classification.

Items	Types	Low-risk group *n* (%)	High-risk group *n* (%)	*N*	*P* values
Gender	Males	53 (29.28%)	20 (11.05%)	73	0.432
	Females	83 (45.86%)	25 (13.81%)	108	
Age	Average age	48 ± 9.81	51 ± 11.39	181	0.873
Physical examination or accidental discovery	Yes	34 (18.78%)	33 (18.23%)	67	0.796
	No	102 (56.35%)	12 (6.63%)	114	
Respiratory tract infection	Yes	9 (4.97%)	9 (4.97%)	18	0.694
	No	127 (70.17%)	36 (19.89%)	163	
Chest distress and shortness of breath	Yes	9 (4.97%)	5 (2.76%)	14	0.671
	No	127 (70,17%)	40 (22.10%)	167	
Chest pain	Yes	5 (2.76%)	4 (2.21%)	9 172	0.856
	No	131 (72.38%)	41 (22.65%)		
Palpitation	Yes	0 (0%)	2 (1.10%)	2	0.316
	No	136 (100%)	43 (23.76%)	179	
Hoarse voice	Yes	2 (1.10%) 134 (74.03%)	1 (0.55%) 44 (24.31%)	3 178	0.210
	No				
	No				
MG	Yes	25 (13.81%)	40 (22.10%)	65	1.000
	No	111 (61.33%)	5 (2.76%)	116	0.107

## Data Availability

The data used to support the findings of this study are available from the corresponding author upon request.
